The article "Incidence and Clinical Outcomes of Hip Fractures Involving Both the Subcapital Area and the Trochanteric or Subtrochanteric Area" was published in 2019. Journal: Adv Orthop.

# Incidence and Clinical Outcomes of Hip Fractures Involving Both the Subcapital Area and the Trochanteric or Subtrochanteric Area

**DOI:** 10.1155/2019/1628683

**Published:** 2019-04-04

**Authors:** Takayuki Tani, Hiroaki Kijima, Natsuo Konishi, Hitoshi Kubota, Shin Yamada, Hiroshi Tazawa, Norio Suzuki, Keiji Kamo, Yoshihiko Okudera, Masashi Fujii, Ken Sasaki, Tetsuya Kawano, Yosuke Iwamoto, Itsuki Nagahata, Naohisa Miyakoshi, Yoichi Shimada

**Affiliations:** ^1^Akita Hip Research Group, Akita 010-8543, Japan; ^2^Department of Orthopedic Surgery, Akita University Graduate School of Medicine, Hondo, Akita 010-8543, Japan

## Abstract

**Purpose:**

Proximal femoral fractures involving both the subcapital area and the trochanteric or subtrochanteric area have rarely been reported, but they are not uncommon. However, few studies have reported the incidence or clinical outcomes of such fractures. This study investigated such fractures.

**Methods:**

In area classification, the proximal femur is divided into 4 areas by 3 boundary planes: the first plane is the center of femoral neck; the second plane is the border between femoral neck and femoral trochanter; and the third plane links the inferior borders of greater and lesser trochanters. A fracture only in the first area is classified as a Type 1 fracture; one in the first and second areas is classified as a Type 1-2 fracture. Therefore, proximal femoral fractures involving both the subcapital area and the trochanteric area are classified as Type 1-2-3, and those involving both the subcapital area and the subtrochanteric area are classified as Type 1-2-3-4. In this study, a total of 1042 femoral proximal fractures were classified by area classification, and the treatment methods and the failure rates were investigated only for Types 1-2-3 and 1-2-3-4 cases. The failure rate was defined as the incidence of internal fixator cut-out or telescoping >10 mm.

**Results:**

Types 1-2-3 and 1-2-3-4 fractures accounted for 1.72%. Surgical treatment was performed for 89%. Of these, 56% underwent osteosynthesis, but the failure rate was 33%. The other patients (44%) underwent prosthetic replacement. Fracture lines of all these fractures were present along trochanteric fossa to intertrochanteric fossa in posterior aspect and just below the femoral head in anterior aspect.

**Conclusion:**

Fracture involving the subcapital area to the trochanteric or subtrochanteric area was found in approximately 2%. In patients for whom prosthetic replacement was selected, good results were obtained. However, 1/3 of patients who underwent osteosynthesis had poor results.

## 1. Introduction

Fractures of the proximal femur are classified into femoral neck fractures, femoral trochanteric fractures, or basicervical fractures. However, fractures rarely involve the subcapital area to the trochanteric or subtrochanteric area [1–3]. Although such fractures are difficult to treat, few studies have investigated the treatment methods and clinical results of these fractures, because almost all classifications of proximal femoral fractures cannot classify these fractures.

The article "Incidence and Clinical Outcomes of Hip Fractures Involving Both the Subcapital Area and the Trochanteric or Subtrochanteric Area" was published in 2019. Journal: Adv Orthop.

The area classification is a comprehensive classification of proximal femoral fractures that facilitates classification based on three-dimensional computed tomography (3D-CT) findings. It is also possible to detect fractures involving the subcapital area to the trochanteric or subtrochanteric region by using this classification. In addition, this classification is reliable and useful for selecting therapeutic strategies [4, 5].

In the area classification, the proximal femur is divided into 4 areas using 3 borders: the center of the femoral neck, the border between the femoral neck and the trochanteric region, and the plane linking the inferior borders of the greater and lesser trochanters. The subcapital area is defined as Area 1, the base of the femoral neck area is defined as Area 2, the trochanteric area is defined as Area 3, and the subtrochanteric area is defined as Area 4. Then, a fracture line that exists only in Area 1 is classified as a Type 1 fracture, and one in Area 1 and Area 2 is classified as a Type 1-2 fracture [5].

Thus, fractures involving the subcapital area to the trochanteric or subtrochanteric area are classified as Type 1-2-3 or Type 1-2-3-4 fractures, in which the fracture line involves an extensive area: Area 1 to Area 3 or Area 4 according to the area classification (Figures 1 and 2).

Therefore, in this study, the incidence, the 3-dimensional features of the fracture lines, and the clinical results of Type 1-2-3 and 1-2-3-4 fractures, which may be markedly unstable and require careful surgery for osteosynthesis, were investigated.

## 2. Subjects and Methods

The subjects were 1,042 patients (209 males, 833 females) with proximal femoral fractures who were treated at 8 general hospitals between January 2014 and December 2015. Their mean age was 82 years (range, 26-108 years). The type of fracture was retrospectively evaluated using the area classification [4, 5] based on X-ray films and 3D-CT images.

Subsequently, patients in whom the type of fracture were evaluated as Type 1-2-3 or 1-2-3-4, which refers to fractures involving the subcapital area to the trochanter or subtrochanteric region based on area classification, were selected, and 3D-CT images were examined from the anterior and posterior sides for all patients.

The article "Incidence and Clinical Outcomes of Hip Fractures Involving Both the Subcapital Area and the Trochanteric or Subtrochanteric Area" was published in 2019. Journal: Adv Orthop.

Furthermore, internal fixation materials used to treat these types of fractures and the presence of lag screw cut-out and ≥10 mm telescoping on the final assessment were investigated. Patients with cut-out or telescoping ≥10 mm of the internal fixator were assigned to the failure group (Group F). The incidence of Group F was defined as the failure rate (F rate).

In addition, when the prosthetic replacement was selected as the treatment for these cases the dislocation or the infection cases were assigned to the failure.

## 3. Results

Of 1,042 patients with fracture of the proximal femur, 18 (1.72%) had a Type 1-2-3 or 1-2-3-4 fracture (278 had Type 1, 235 had Type 2-3, 227 had Type 3, 100 had Type 1-2, 87 had Type 3-4, 66 had Type 2-3-4, 17 had Type 4, 10 had Type 2, and 4 cases were unclear). The average follow-up period is 5.4 months (1-18 months).

In 17 of the 18 patients, fracture lines on 3D-CT were present along the trochanteric fossa to the intertrochanteric fossa in the posterior region and the subcapital area in the anterior region (Figure 2).

Of these, conservative treatment was performed for 2 (11%), and surgical treatment was selected for the other 16 (89%). Of the 16 patients, osteosynthesis was selected for 9 (56%) (Figure 3). Of these, a short femoral nail (SFN) was used in 5 (56%), a compression hip screw (CHS) was used in 3 (33%), and a long femoral nail was used in 1 (11%). Of the 5 SFN-treated patients, the use of two lag screws was selected for 3 (60%). Of the 3 CHS-treated patients, the use of two lag screws was selected for 2 (67%), whereas an antirotation screw was added in 1 (33%) (Figure 4).

Of the 9 patients treated by osteosynthesis, ≥10 mm lag screw telescoping was observed in 3 (33%); thus, the F rate was 33%. Of the 3 patients, an SFN with a single lag screw was used in 1, an SFN with two lag screws was used in 1, and a CHS with two lag screws was used in 1. Cut-out of the internal fixator was not observed in this study.

For the remaining 7 patients (44%), prosthetic replacement (femoral head replacement) was selected, and there was no failure in any patient with prosthetic replacement.

## 4. Discussion

Fractures involving the subcapital area to the trochanteric or subtrochanteric region are impossible to classify other than by Area classification of proximal femoral fractures. Therefore, it is impossible to survey the results of treatment for fractures involving the subcapital area to the trochanteric or subtrochanteric region without using the area classification. This study is the first to investigate the incidence, courses of fracture lines, and clinical results of fractures involving the subcapital area to the trochanteric or subtrochanteric region using area classification.

The article "Incidence and Clinical Outcomes of Hip Fractures Involving Both the Subcapital Area and the Trochanteric or Subtrochanteric Area" was published in 2019. Journal: Adv Orthop.

In the present study, such fractures were found in 1.72% of all proximal femoral fractures. Furthermore, the survey using 3D-CT images showed that the fracture lines were present along the trochanteric fossa to the intertrochanteric fossa in the posterior aspect and the subcapital area in the anterior aspect in almost all patients. Of patients who underwent osteosynthesis, more than 30% had poor results.

Most fractures of the proximal femur can be classified as cervical/trochanteric fractures. Regarding the respective types of fractures, several classifications, such as the AO/OTA classification, have been used. However, in some patients, a continuous fracture line involving the area just below the femoral head to the trochanteric or subtrochanteric region is present, extending over the border of classification. These fractures are impossible to classify other than by area classification. Such fractures have been reported as “simultaneous ipsilateral or rare fractures”, but a consensus regarding imaging findings, appropriate treatment, or treatment results has not been reached [1–3, 6, 7].

In this study, proximal femoral fractures were evaluated using 3D-CT in more than 1,000 patients, and the incidence of fracture involving the subcapital area to the trochanteric or subtrochanteric region (area classification Type 1-2-3 or 1-2-3-4) was approximately 2%, indicating that this type of fracture frequently causes postosteosynthesis complications.

In almost all patients, fracture lines were present along the trochanteric fossa to the intertrochanteric fossa in the posterior aspect and below the femoral head proximal to the intertrochanteric line (area classification: Area 1) in the anterior aspect. Briefly, in the posterior aspect, the fracture line was consistent with that of a trochanteric fracture, and in the anterior aspect, it was consistent with that of a cervical fracture. According to a recent study that examined basicervical femoral fracture using 3D-CT, it is a subtype of trochanteric fracture in which the fracture line in the posterior cervix is consistent with that of a trochanteric fracture, whereas that in the anterior cervix differs [8]. This is consistent with the fracture lines observed in the present study.

Since a basicervical fracture is similar to a trochanteric fracture in blood supply for femoral head, osteosynthesis is frequently selected. However, previous studies reported a high incidence of complications related to instability [9–11]. In this study, more than 30% of patients who underwent osteosynthesis had poor results. On the other hand, the results of prosthetic replacement were good.

The article "Incidence and Clinical Outcomes of Hip Fractures Involving Both the Subcapital Area and the Trochanteric or Subtrochanteric Area" was published in 2019. Journal: Adv Orthop.

One limitation of this study is that the therapeutic strategies were not standardized among institutions. Therefore, details regarding cases in which osteosynthesis were possible, whether internal fixation materials appropriate for osteosynthesis were used, and procedure-related limitations were not obtained. However, in the future, an optimal strategy to treat fractures involving the subcapital area to the trochanteric or subtrochanteric region may be selected by classifying proximal femoral fractures using area classification and focusing on Type 1-2-3 or 1-2-3-4 fractures through continued surveys. This study presents important findings for this purpose.

## Figures and Tables

**Figure 1:** Type 1-2-3 fractures involving the area below the femoral head (area classification: Area 1) to the trochanteric area (Area 3) and Type 1-2-3-4 fractures involving Area 1 to the subtrochanteric area (Area 4).

**Figure 2:** Anterior fracture line and posterior fracture line of Type 1-2-3-4 fractures. Fracture lines are present along the trochanteric fossa to the intertrochanteric fossa in the posterior region and below the femoral head in the anterior region.

**Figure 3:** Of 1,042 patients with fracture of the proximal femur, Type 1-2-3(-4) fractures account for 1.72%, with osteosynthesis performed for 56% and prosthetic replacement performed for 44%.

**Figure 4:** Of patients who underwent osteosynthesis for Type 1-2-3(-4) fractures, treatment consisted of a short femoral nail with single lag screw in 22%, a short femoral nail with double lag screw in 33%, a compression hip screw with double lag screw in 22%, a compression hip screw with antirotation screw in 11%, and a long femoral nail in 11%.

## Data Availability

The data that support the findings of this study are available from the corresponding author, upon reasonable request.
